# Long non-coding RNA CCL2 promoted gastric cancer function via miR-128/ PARP2 signal pathway

**DOI:** 10.1080/21655979.2021.2020548

**Published:** 2022-01-08

**Authors:** Liang Ma, Yunshan Jiang, Ning Wu

**Affiliations:** a Department of Digestive Internal Medicine,Shaoxing No. 2 Hospital Medical Community General Hospital,Shaoxing, Zhejiang Province, China; b Department of Oncology, Longyan First Hospital, Affiliated to Fujian Medical University,Longyan, P.R. China; c Department of Oncology, Shanghai Pudong New Area Gongli Hospital, Shanghai, P.R. China

**Keywords:** Gastric cancer, invasion, PARP2, proliferation, miR-128, CCL2, migration

## Abstract

Amounts of studies have revealed long non-coding RNA (lncRNA) was related to the development of gastric cancer. Here, our results suggested the function and regulatory mechanism of CCL2 in gastric cancer. Quantitative polymerase-chain reaction (qPCR) was employed to inspect lncRNA CCL2 and miR-128 expression in normal gastric cell line (GES-1) and tumor cell lines (HGC-27 and MKN-45). The effects of CCL2 and miR-128 were measured via Luciferase reporter test. Western blot was used to check PARP2 protein expression. CCL2 expression and PARP2 protein levels were up-regulated, while miR-128 expression was obviously lower. Meanwhile, CCL2 down-regulating significantly repressed the proliferation, migration, and invasion by regulating miR-128. In addition, we proved miR-128 was a direct target of CCL2 through double luciferase assay and bioinformatics analysis. Moreover, miR-128 markedly inhibited the proliferation, migration, and invasion in gastric cancer. More importantly, miR-128 could reverse the effects of lncRNA CCL2 knocked down. PARP2-si obviously suppressed in gastric cancer proliferation, migration, and invasion. Meanwhile, miR-128 mimic and the knockout of CCL2 distinctly decreased PARP2 protein level. Additionally, luciferase report experiments certificated that PARP2 targeted miR-128, implying PARP2 directly interacted with miR-128 in gastric cancer. More interestingly, the downregulation of PARP could reverse the trend triggered by miR-128 inhibitor in gastric tumor. All over these results showed lncRNA CCL2 played importance of role in gastric tumor via miR-128/PARP2 axis signal pathway. LncRNA CCL2 accelerated gastric cancer progression by regulating miR-128/PARP2 signaling pathway, providing a novel possible strategy for the treatment of gastric cancer.

## Introduction

Gastric cancer is a kind of epidemic and highly invasive malignant tumors [1–5]. Its occurrence and development are as sudden as other tumors [6]. Usually, changes in cell growth regulation and patterns lead to alter in precancerous lesions and related genes [7–9]. *Helicobacter pylori* infection, smoking, and obesity were considered to be the most common causes of gastric cancer [10]. Therefore, we should have a deeper understanding of the occurrence and development mechanism of gastric cancer and adopt more effective treatment strategies [11].

LncRNA has become a research hotspot [12,13] and it not only participates in cell cycle, differentiation, apoptosis, senescence, cytoplasmic, or nuclear plasma transport but also has important biological functions such as epigenetic and transcriptional regulation and translation regulation [14,15]. LncRNA RHPN1-AS1 knockout depressed glioma cells proliferation, migration, and invasion via miR-625-5P/REG3A [16]. ZFAS1 expression was related to the progress of PTC through microRNA-590-3P/HMGA2 aixs [17]. A large number of studies have shown that lncRNAs played indispensable role in the process of gastric cancer [18,19]. LncRNA SNHG3 promoted gastric cancer progression by MED18 genes methylation [20]. LncRNA SNHG1 could regulate DNMT1 to further promote the proliferation of gastric cancer [21]. Wei [22] believed that LNCRNA MEG3 could reduce the proliferation and metastasis of gastric cancer by increasing P53 expression. In the study of Jason E. Fish, lncRNA CCL2 regulated CCL2 expression in human vascular endothelial cells, which may contribute to the formation of atherogenesis [23]. However, there are rare studies on the biological function and molecular mechanism of CCL2 in gastric cancer.

Given the important role of lncRNAs, especially CCL2 in cancer, we postulated that it also promotes the oncogenic function of gastric cancer cells. As both miR-128 and PARP2 play critical roles in gastric cancer [24,25], we hypothesized that CCL2 could sponge miR-128, thereby potentially regulating PARP2. The purpose of this study was to explore the mechanism of miR-128/PARP2 signaling pathway mediated by lncRNA CCL2 in gastric cancer, and to propose a novel perspective for gastric cancer treatment.

## Methods

### Cell culture and treatment

GES-1 (epithelial cells derived from human gastric mucosa), MKN-45 and HGC-27 (CelBio, China) were cultured in RPMI medium containing 10% fetal bovine serum (Gibco, Ma, USA) and 5% CO_2_ at 37°C humidified incubator containing.

### SiRNA transfection

Sh-CCL2, PARP2-si, miR-128 mimics, and miR-128 inhibitor were designed and synthesized by GenePharma (Shanghai, China). Cells were transfected with transfection reagent Lipo3000 follow the reagent instructions (Invitrogen, Arlsbad, CA, USA) for 4 hours and then replaced with normal medium. After 48 hours of treatment, QPCR and Western blot were employed to detect the transfection efficiency.

### Luciferase reporter test

HEK293T cells inoculated on 96-well plate were co-transfected with 50ng miR-128 plasmid or control plasmid with 90ng CCL2 3’-UTR-WT or CCL2 3’-UTR-Mut by lipo 3000 (Invitrogen, Arlsbad, CA, USA). After 48 hours, cells were collected in accordance with double luciferase assay (Promega, Madison, WI, USA). MiR-128, plasmid, luciferase structure, CCL2 3’-UTR or 3’-UTR-Mut were purchased from Gene Pharmaceutical (Shanghai) Co., Ltd.

### Cell counting kit-8 assays

Transfected cells were inoculated into 96-well plate culture medium. Then, 10 μL CCK-8 (CK04, Kumamoto, Japan) was added and incubated for 3 hours at the designated time point after transfection. Finally, the absorbance is tested by a microplate reader (9200, BioRad Laboratories, CA, USA) at 450 nm.

### Transwell assay

Cells in 200 μl of serum-free Roswell Park Memorial Institute-1640 were inoculated into the upper chambers, and 10% fetal bovine serum was added to the lower transwell chambers (Biosciences, Franklin Lakes, USA). After incubation at 37°C for 48 hours, the cells on the upper side of the membrane were removed with cotton swabs. Cells immobilized on the lower surface were fixed with 100% precooled methanol and fixed with 0.1% crystal violet. The same experimental procedure was performed for cell invasion test except for transwell cell (Corning, toxbury, Massachusetts, USA).

### Real time PCR

RNA was isolated using trizol reagent (Cwbio, China) and primescript RT Kit (Perfect real time) (Takara, Japan) was employed to cDNA synthesis following to manufacturer’s information. PCR was executed using iTaqTM universal SYBR®Green Supermix (Bio-Rad, Hercules, CA). Primer sequences involved are summarized in Table 1. PCR reactions containing SG (SYBR® Green) were optimized using Promega’s TaqDNA polymerase after the primers were dissolved. The reaction was performed using reverse transcriptase (Promega) to reverse transcribe the sample RNA into cDNA. For relative quantification, PCR amplification of the target gene and housekeeping gene of the sample is required, and gradient dilution of the product is used for the standard curve. The standard curve sample and the test sample were added into the RealTime PCR reaction solution containing SG (TaqBeadTM hot-start polymerase was from Promega Company), respectively. For real-time PCR amplification and detection. The test results were analyzed by standard curve to quantify the target genes of the tested samples.

**Table 1.** Sequences used for QPCR

Name	sequences
LncRNA-CCL2 F	GGGAGACTGAGGCCATGAAC
LncRNA-CCL2 R	GCTTTGCCAAGTCACTTCCC
miR-128 F U6 F U6 R GAPDH-F GAPDH-R	UCACAGUGAACCGGUCUCUUU TGCGGGTGCTCGCTTCGCAGC AGCGGGGGAAGTGACGCAGTC GATTCCACCCATGHCCAAATTC CTGGAAGATGGTGATGGGATT

### Western blot analysis

Ten percent SDS-PAGE gel and immobilon®PVDF membranes (Merck KGaA, Darmstadt, Germany) were used to fractionate cellular proteins. Blocked with 5% skimmed milk, membranes were developed overnight at 4°C with primary antibodies against PARP2 (1:1000, Cell signaling tech), β-actin (1:1000, Cell signaling tech). After incubation with the second antibody binding to HRP (goat anti-rabbit IgG, Proteintech, China), the enhanced chemiluminescence detection kit (Cwbio, Beijing, China) was used to develop the membrane and the gel imaging system was used to detect the results.

### Statistical analysis

All results were shown as mean ± SD. Two-way ANOVA and student *t*-test were performed with GraphPad Prism 6 (GraphPad Software, San Diego, CA). P < 0.05 was considered statistically significant.

## Results

### LncRNA CCL2 downregulation distinctly suppressed gastric cancer cells function

LncRNA plays an important role in gastric cancer progression. It serves as a sponge for a lot of miRNAs and decrease the level of them and thereby exerting inhibitory or conducive effects on cellular proliferation, invasion, and migration.

Compared with GES-1, CCL2 expression was obviously upregulated in HGC-27 and MKN-45 cells (Figure 1a). Then, the expression of CCL2 was sharply down-regulated compared with the negative control group after sh-CCL2 treatment and CCL2 transfection efficiency was tested using real-time PCR (Figure 1b). Meanwhile, CCK-8 and transwell assays were employed to investigate the function of gastric cancer cells. All in all, results suggested that CCL2 knocked down by sh-CCL2 prominently curbed the proliferation (Figure 1c and 1d), invasion (Figure 1e) and migration (Figure 1f) of gastric cancer.

**Figure 1.** **LncRNA CCL2 downregulation distinctly suppressed gastric cancer cells function. a** LncRNA CCL2 expression in MKN-45 and HGC-27 cells was measured by QPCR. **b** LncRNA CCL2 expression in MKN-45 and HGC-27 cells was measured by QPCR. **c-d** CCK-8 assay was employed to detect cell proliferation after transfection with sh-lncRNA CCL2. **e** Transwell assay was employed to detect cell invasion after transfection with sh-lncRNA CCL2. **f** Transwell assay was employed to detect cell migration after transfection with sh-lncRNA CCL2. The data were showed as mean ± SD. n = 3 *p < 0.05.

### LncRNA CCL2 directly inhibited miR-128 expression and miR-128 is lower

As it is proved that lncRNA CCL2 promotes proliferation, invasion, and migration of gastric cancer cells, it is imperative to find out the target miRNAs and underlying mechanism.

To study the mechanism of CCL2 in the occurrence and development of gastric cancer, bioinformatics analysis software was used to predict the potential targeting miRNAs of CCL2. As a result, miR-128 was a potential regulator of CCL2 (Figure 2a). Additionally, the double luciferase report experiment showed that the miR-128 mimic significantly reduced the luciferase activity of CCL2-WT reporter and the luciferase activity of CCL2-MUT reporter did not decrease obviously in HEK293T cells (Figure 2b). We further confirmed the effect of CCL2 on miR-128 expression and results showed miR-128 expression transfected with sh-CCL2 prominently increased (Figure 2c). Meanwhile, miR-128 expression evidently decreased (Figure 2d). Taken together, results showed that CCL2 inhibited miR-128 expression through direct interaction in gastric cancer.

**Figure 2.** **LncRNA CCL2 directly inhibited miR-128 expression and miR-128 is lower. a** The predicted miR-128 binging sites in lncRNA CCL2. **b** Effect of miR-128 on the activity of lncRNA CCL2 reporter luciferase was checked by luciferase assay. **c** miR-128 expression was determined after transfection with sh-lncRNA CCL2 by QPCR. **d** miR-128 expression was measured by QPCR. The data are indicated as mean ± SD. n = 3. *p < 0.05.

### MicroRNA-128 clearly inhibited the function of HGC-27 and MKN-45 cells

Given the evidence showing that miRNA-128 could be targeted by CCL2 using HEK293T cells as a tool, we would like to further investigate the function of miRNA-128 in HGC-27 and MKN-45 cells.

Based on the conclusion of the appeal, we further explore whether microRNA-128 was involved in the occurrence and development of gastric cancer. Our study stated miR-128 mimic obviously elevated the expression of miR-128 compared with the negative control group and the transfection efficiency of miR-128 was checked by qPCR (Figure 3a). Additionally, our results certificated that miR-128 mimic extremely inhibited cell proliferation, migration, and invasion (Figure 3b-e). Conversely, miR-128 inhibitors obviously caused the opposite trend on cell proliferation, migration, and invasion (Figure 3f-i).

**Figure 3.** **MicroRNA-128 clearly inhibited the function of HGC-27 and MKN-45 cells. a** MiRNA-128 expression was increased after miRNA-128 mimic treatment by QPCR. **b-c** The cell proliferation after miRNA-128 mimic treatment was measured by CCK-8 assay. **d-e** transwell assay was used to detected invasion and migration after miRNA-128 mimic treatment. **f-g** CCK-8 assay was used to detected cell proliferation after miRNA-128 inhibitor treatment. **h-i** Transwell assay was used to detected cell proliferation after miRNA-128 inhibitor treatment. The data are showed as mean ± SD. n = 3. *p < 0.05.

### MiR-128 reversed the effects of silencing of CCL2 in gastric cancer cells

As the inhibitory function of miR-128 in HGC-27 and MKN-45 cells has been exemplified, the interaction between CCL2 and miR-128 shall be further verified in gastric cell lines. To further probe into whether the role of CCL2 in the progression of gastric cancer was mediated by miR-128, miR-128 inhibitor was transfected into cells transfected with sh-CCL2. Results stated that the reduction of sh-CCL2 induced on proliferation (Figure 4a and 4b), invasion (Figure 4c) and migration (Figure 4d) was significantly increased by the knockout of microRNA-128. Altogether, these data suggested that CCL2 partially plays a carcinogenic role by inhibiting miR-128 expression.

**Figure 4.** **MiR-128 reversed the effects of silencing of CCL2 in gastric cancer cells. a-b** The cell proliferation after transfection with sh-NC or sh-lncRNA CCL2 along with miR-128 inhibitor was measured using CCK-8 assay. **c-d** transwell assay was employed to detected invasion and migration after transfection with sh-NC or sh-lncRNA CCL2 along with miR-128 inhibitor. The data are showed as mean ± SD. n = 3. *p < 0.05.

### MiR-128 directly suppressed PARP2 protein level

PARP2 is a main member of PARP family, which has many biological functions, including DNA repair, synthetic lethality, apoptosis, necrosis, histone binding, and so on. To make clear whether miR-128 was directly mediated by PARP2 in gastric cancer. Therefore, miR-128 mimics was transfected into cells and PARP2 protein level was investigated. Results showed that miR-128 mimic resulted in an obvious decrease in PARP2 expression and converse results were found when silencing miR-128 (Figure 5a and 5b). luciferase assay and bioinformatics analysis indicated PARP2 was a potential target of miR-128 (Figure 5c and 5d). In addition, PARP2 level was clearly cut down by sh-CCL2 (Figure 5e). Meanwhile, PARP2 expression was up-regulated in HGC-27 and MKN-45 (Figure 5f). In general, CCL2 employed a key role in gastric cancer progression via regulating miR-128/PARP2 signaling pathway.

**Figure 5.** **MiR-128 directly suppressed PARP2 protein level. a-b** PARP2 protein level was investigated by Western blot. **c** The predicted miR-128 binging sites in PARP2. **d** Effect of miR-128 on the activity of PARP2 reporter luciferase was checked by luciferase assay. **e-f** Western blot was employed to detected PARP2. The data are expressed as mean ± SD. n = 3. *p < 0.05.

### PARP2 down-regulation repressed cells function of gastric cancer

As the direct interaction has been proved by luciferase reporter experiment, we assumed that PARP2 could promote the cellular proliferation, invasion, and migration of gastric cancer. To further investigate the regulatory mechanism of PARP2 in gastric cancer, PARP2 expression was distinctly suppressed by si-PARP2 (Figure 6a). Then, we tested the change on proliferation, migration, and invasion after si-PARP2 treatment. Results indicated that down-regulated PARP2 clearly restrained cell proliferation, migration, and invasion (Figure 6b-e). The above experimental data showed that CCL2 was involved in gastric cancer progression through possibly regulating miRNA-128/PARP2.

**Figure 6.** **PARP2 down-regulation repressed cells function of gastric cancer. a** PARP2 was tested after PARP2-si treatment by Western blot. **b-c** The cell proliferation after PARP2-si treatment was checked by CCK-8 assay. **d-e** Cell invasion and migration after PARP2-si treatment were measured using transwell assay. The data are indicated as mean ± SD. n = 5. *p < 0.05.

### PARP2 reversed the effects of niR-128 inhibitor in gastric cancer cells

We further make clear whether the regulation of miRNA-128 was medicated by PARP2 on gastric cancer. miR-128 inhibitor and PARP2-si were co-transfected into MKN-45 and HGC-27 cells and result indicated the knockdown of PARP2 extremely reversed miR-128 inhibitor effect of proliferation (Figure 7a-b), migration, and invasion (Figure 7c-d). Collectively, these data clearly suggested that CCL2 played a carcinogenic role by regulating miRNA-128/PARP2 signal pathway, indicating that targeting CCL2/miRNA-128/PARP2 may be a new effective strategy for gastric cancer therapy.

**Figure 7.** **PARP2 reversed the effects of niR-128 inhibitor in gastric cancer cells. a-b** The cell proliferation after co-transfection with miR-128 inhibitor and PARP-si was detected using CCK-8 test. **c-d** Invasion and migration of MKN-45 and HGC-27 cells after co-transfection miR-128 inhibitor and PARP-si were measured by transwell assay. The data are expressed as mean ± SD. n = 3. *p < 0.05.

## Discussion

More and more evidence suggested that lncRNAs have an importance of role in gastric cancer progression. Peng K etl stated PART-1 targeted TGFBR2/Smad3 to regulate chondrocytes function via miR-590-3p in osteoarthritis [24]. LncRNA CCL2 was highly expressed in atherosclerotic and acted as a powerful predictor of prognosis. Therefore, our study discussed its role in gastric cancer. Our research suggested CCL2 was significantly elevated in gastric cancer and the knockdown of CCL2 markedly suppressed gastric cancer cell function. These results suggested that CCL2 may play an oncogene role in gastric cancer and the knockout of CCL2 was beneficial to reduce the occurrence and development of gastric cancer.

Amounts of studies have previously been uncovered the importance of miRNAs in regulating the development of gastric cancer [25–27]. Such as miR-331 could inhibited gastric cancer development by targeting MSI1 and it could be used as a predictor and prognostic indicator of gastric cancer [28]. MiRNA imbalance contributed to the progress of gastric cancer [29,30]. Smurf1, as an anticancer agent, could be removed from DDP-resistant gastric cancer [31,32–35]. MiR-128 was related to the regulation of various cancer [30,31], but the specific mechanism of its involvement in gastric cancer was still not known. In our study, luciferase assay and bioinformatics analysis showed miR-128 was a direct target of CCL2 and CCL2 down-regulating evidently increased miR-128 expression. Further experiments indicated microRNA-128 expression was prominently lower. Additionally, microRNA-128 overexpression extremely inhibited cell proliferation, migration, and invasion, whereas microRNA-128 silence caused the opposite result. Moreover, miR-128 inhibitor could partly reverse the regulatory effects of downregulation of CCL2. Based on the above findings implied that CCL2 played key role in gastric cancer through miR-128 and miR-128 may function as a gastric cancer inhibitor.

PARP enzymes have various biological function such as transcriptional regulation, maintenance of genomic stability, energy metabolism, and cell death. Poly PARP2 is a member of PARP family having varied biological functions: apoptosis, necrosis, and so on. In our study, PARP2 protein level in gastric cancer was remarkably higher and miR-128 mimic dramatically suppressed PARP2 expression at protein level in MKN-45 and HGC-27 cells. PARP2 protein was substantially reduced after treatment with sh-CCL2. Meanwhile, luciferase report test conformed PARP2 was a direct target of miR-128 and the down-regulation of PARP2 resulted in clearly decrease cell proliferation, migration, and invasion. More importantly, PARP down-regulation could reverse the effect induced by miR-128 inhibitor treatment, implying PARP2 directly regulated miR-128 during gastric cancer development. Above results suggested that CCL2/miR-128/PARP2 axis signal pathway played indispensable role in the occurrence and development of gastric cancer, which provided a theoretical basis of clinical application for gastric cancer.

## Conclusion

As far as we know, our study was the first to reveal high levels of CCL2 and discover new function for CCL2 in gastric cancer. We also raised a novel mechanism of direct interaction between CCL2 with miR-128 and miR-128 with PARP2, implying lncRNA CCL2 could regulate gastric cancer through miR-128/PARP2. These findings further deepen our understanding of the pharmacological effects of CCL2 and provided new information for further elucidation of its mechanism. It is helpful to better understand the molecular mechanism of the progression of gastric cancer and provided a new potential strategy for gastric cancer treatment.

## Research highlight

1. This study demonstrated the role and underlying mechanism of long non-coding RNA CCL2 in gastric cancer.
2. It revealed the association between CCL2 and 2 critical components in the oncogenesis of gastric cancer: miR-128 and PARP2
3. It provided direct evidence for the interaction between CCL2 and miR-128/PARP2 axis
